# Comparison of the Efficacy and Safety of Neuroendoscopic Endonasal Transsphenoidal Surgeries and Intracranial Endoscopic Pterional Approach in Resection of Tuberculum Sellae Meningiomas

This article has been retracted.

**DOI:** 10.1155/2022/4542815

**Published:** 2022-06-07

**Authors:** Zhenrong Lin, Ziyue Wu, Yuzhe Wang, Weiwei Wang, Weixin Zheng, Ruisheng Lin, Aishun Guo

**Affiliations:** ^1^Department of Neurosurgery, Zhangzhou Affiliated Hospital of Fujian Medical University, Zhangzhou, Fujian 363000, China; ^2^Department of Nephrology, Zhangzhou Affiliated Hospital of Fujian Medical University, Zhangzhou, Fujian 363000, China; ^3^The Third Clinical Medical College, Fujian Medical University, Fuzhou, Fujian 350001, China; ^4^The Graduate School of Fujian Medical University, Fuzhou, Fujian 350001, China

## Abstract

**Objective:**

To compare of the efficacy and safety of neuroendoscopic endonasal transsphenoidal surgeries and intracranial endoscopic pterional approach in resection of tuberculum sellae meningioma.

**Methods:**

From January 2014 to June 2021, 60 patients with tuberculum sellae meningioma diagnosed and treated in our hospital were enrolled and randomly divided into study group and control group. The tuberculum sellae meningioma was removed by neuroendoscopic endonasal transsphenoidal surgeries in the study group, while the intracranial endoscopic pterional approach was used in the control group. The chi-square test was used to compare the differences of tumor complete resection rate, visual acuity improvement rate, total effective rate at 3 months after operation, and adverse reactions between the two groups.

**Results:**

The clinical characteristics of the two groups were comparable (*P* > 0.05). After surgical treatment, the complete resection rate in the study group was higher than that in the control group (93.3% vs 70.0%), and the difference was statistically significant (*P*=0.020). After treatment, the visual acuity improvement rate of the study group was 83.3% (25/30), which was significantly higher than that of the control group (60.0%, 18/30), and the difference was statistically significant (*χ*^2^ = 4.022, *P*=0.045). After surgical treatment, the total effective rate at 3 months after operation was higher in the study group than in the control group (96.7% vs 83.3%), with statistical significance (*P*=0.041). There was no significant difference in postoperative adverse reactions between the study group and control group (33.3% vs 30.0%, *P*=0.781).

**Conclusion:**

The neuroendoscopic endonasal transsphenoidal surgeries has significant efficacy and can significantly improve the visual acuity of patients without increasing adverse reactions, which is worthy of clinical promotion.

## 1. Introduction

Meningioma is a common intracranial tumor, with tuberculum sellae meningioma (TSM) accounting for about 3% to 10% of intracranial meningiomas [1]. Compared with other meningiomas, tuberculum sellae meningioma has its specificity in clinical manifestations, epidemiological characteristics, and pathological and anatomical features. Tuberculum sellae meningioma often refers to meningioma originating from tuberculum sellae, optic chiasma, and diaphragm sellae, which can damage optic chiasma and optic nerve, causing progressive visual and visual field disorders. The larger tumor may be accompanied by headache, epilepsy, etc., and abnormal secretion of endocrine hormones may occur when the pituitary gland is affected [2]. Tuberculum sellae meningiomas are more common in adults, mainly between 45 and 55 years old, with more women than men, and the incidence of women is twice as high as that of men [3]. Tuberculum sellae meningioma usually has a deep location and complex anatomical structure, which is close to important tissues such as optic nerve, optic chiasm, internal carotid artery, and pituitary gland. Therefore, it is difficult to operate and the surgical effect is not ideal [4]. Therefore, how to improve the visual acuity of patients and improve the therapeutic effect is the focus and difficulty of current surgical treatment. In recent years, with the rapid development of neurology and microsurgery, surgical treatment methods are also being explored [5]. Intracranial endoscopic pterional approach is the standard method for the treatment of tuberculum sella meningioma. However, there are some problems such as unsatisfactory tumor total resection rate, more traction damage to brain tissue after operation, long operation time, larger wound surface, and various postoperative complications except cerebrospinal fluid leakage [6]. At present, many neurosurgeons are also using neuroendoscopic endonasal transsphenoidal surgeries for the treatment of tuberculum sellae meningioma, which has certain advantages over the traditional approach in the treatment effect, with a higher vision improvement rate and total tumor resection rate [7]. However, there are few studies comparing the therapeutic effects and adverse reactions of neuroendoscopic endonasal transsphenoidal surgeries and intracranial endoscopic pterional approach for tuberculum sellae meningioma resection. In this study, the value of the two surgical methods in the treatment of tuberculum sellae meningioma was compared by comparing the tumor complete resection rate, visual acuity improvement rate, total effective rate at 3 months after operation, and adverse reactions.

## 2. Patients and Methods

### 2.1. Patients

From January 2014 to June 2021, 60 patients with tuberculum sellae meningioma diagnosed and treated in the Zhangzhou Affiliated Hospital of Fujian Medical University were collected, all of which met the diagnostic criteria for tuberculum sellae meningioma. Inclusion criteria are as follows: (1) ≥18 years old; (2) based on the clinical manifestations, endocrine tests, skull MRI, and other typical imaging findings, the patient met the diagnostic criteria for tuberculum sellae meningioma [8]; (3) understand the treatment plan and agree to surgical treatment. Exclusion criteria are as follows: (1) patients with cataracts, glaucoma, and other diseases that can affect vision; (2) serious organ dysfunction such as heart, liver, or kidney; (3) those who have mental disorder and cannot cooperate with the operation, or have contraindications due to other reasons. Patients or authorized family members were informed and signed the consent. The study was approved by the Medical Ethics Committee of Zhangzhou Affiliated Hospital of Fujian Medical University (No. ZA12213). Patients' age, sex, duration of visual impairment, duration of headache, past medical history, drug history, tumor diameter, and relationship between tumor and optic nerve and optic chiasma were analyzed.

### 2.2. Patient Grouping and Treatment Methods

Sixty patients were randomly divided into the study group and control group with 30 patients in each group by the random number table method. Meningiomas of tuberculum sellae were removed by neuroendoscopic endonasal transsphenoidal surgeries in the study group, and intracranial endoscopic pterional approach in the control group. Neuroendoscopic endonasal transsphenoidal surgeries: the patient is supine, and the head is adjusted so that the surgeon's eyes are in line with the patient's nostrils and eyes. The operation is divided into four stages: (1) nasal stage: the nasal mucosa was contracted, the sphenoid sinus opening was found, and the nasal septum with pedicled mucosal flap was made. (2) Sphenoid sinus stage: the bony structure of the anterior wall of the sphenoid sinus was fully exposed to expand the surgical field of vision, and the superior intercavernous sinus was separated by electric coagulation. (3) Tumor resection stage: electrocoagulation excised the basal dura of the tumor, exposed the tumor, and sharply separated the tumor boundary. If the optic canal is invaded, the dural membrane of the optic canal should be opened and cut up. Adequate attention was paid to the protection of the surrounding anatomical structure, electrocoagulation was performed, and the tumor supplying artery was severed. (4) Sellar base reconstruction: three layers of artificial meningeal patch, autogenous fascia lata, and pedicled mucosal flap were used for skull base reconstruction. Iodoform yarn strips or balloons were used to support the structure.

Intracranial endoscopic pterional approach: the patient was placed in the supine position with the head above the heart level. Pterional based on facial structure was identified. Cerebrospinal fluid was released to reduce intracranial pressure, protecting the brain surface was paid attention to, and the frontal lobe straight to the tuberculum sellae was raised to expose the tumor. Electrocoagulation of tumor base was performed to block the tumor blood supply. Electric coagulation was applied to the base of the skull to separate the attachment between the tumor and the dura mater, and the arachnoid membrane around the tumor was sharply separated to fully protect the anatomical structure around the tumor. Mass excision of the tumor was performed. The head is closed after hemostasis.

### 2.3. Observation Indicators

The following indicators were evaluated to observe the postoperative efficacy and adverse reactions. (1) Tumor resection degree and visual acuity improvement: postoperative head MRI was reviewed, and symptom improvement of patients was followed up to evaluate the tumor resection degree and visual acuity improvement. The improvement of visual acuity was assessed by asking the patient's symptoms and examined by the visual acuity scale. (2) Treatment effect 3 months after surgery: significant effective was defined as visual impairment, head ache, and other symptoms basically disappeared; tumor was completely removed, and daily life and work could be resumed. Effective was defined as relief of symptoms such as visual impairment and headache, and improved ability to participate in activities or work. Inefficacy was defined as no improvement in symptoms and signs. Total effective rate = (significant effective + effective)/total number of cases × 100%. (3) Adverse reactions: postoperative adverse reactions were recorded, including anosmia, headache, intracranial infection, and cerebrospinal fluid leakage.

### 2.4. Statistical Analysis

Statistical analysis was performed using the IBM SPSS 22.0 software. The categorical variables were expressed as *n* (%) and compared by the chi-square test. Continuous variables were expressed as mean ± standard deviation and compared with *t*-test. The chi-square test was used to compare the differences of tumor complete resection rate, visual acuity improvement rate, total effective rate at 3 months after operation, and incidence of adverse reactions between the two groups. Bilateral *P* < 0.05 was defined as statistically significant.

## 3. Results

### 3.1. General Data and Clinical Features of Patients

A total of 60 patients with tuberculum sellae meningioma were enrolled in this study. The mean age of patients in the study group was (54.8 ± 9.8) years, and the proportion of males was 50.0% (15/30). The duration of visual impairment and headache was (15.7 ± 4.3) months and (5.5 ± 3.7) months, respectively. Systolic and diastolic blood pressure in the study group were (133.8 ± 13.9) mmHg and (87.7 ± 12.6) mmHg. In the study group, the average tumor diameter was (2.6 ± 0.5) cm, and the proportion of tumor squeezing optic chiasma was 20% (6/30). In the study group, the relationship between meningioma and optic nerve were elation, adhesion, and circumference, respectively, with 46.7% (14/30), 20.0% (6/30), and 33.3% (10/30), respectively. In the control group, the mean age was (56.8 ± 8.2) years and 30.0% (9/30) were males. The duration of visual impairment and headache was (15.1 ± 4.0) months and (5.7 ± 3.5) months, respectively. The proportion of patients with previous hypertension, diabetes, and coronary heart disease in control group was 53.3% (16/30), 33.3% (10/30), and 13.3% (4/30), respectively. In the control group, the average tumor diameter was (2.7 ± 0.3) cm, and the proportion of tumor squeezing optic chiasma was 30.0% (9/30). In the control group, the relationship between meningioma and optic nerve was elation, adhesion, and circumference, respectively, with 43.3% (13/30), 26.7% (8/30), and 30.0% (9/30). The above characteristics were equally comparable between the two groups (*P* > 0.05, Table 1).

### 3.2. The Patient's Tumor Resection

After surgical treatment, the total tumor resection rate was 93.3% (28/30) in the study group and 70.0% (21/30) in the control group. The total resection rate in the study group was significantly higher than that in the control group (*χ*^2^ = 5.455, *P*=0.020) (Table 2).

### 3.3. Improvement of Vision

After surgical treatment, the total visual acuity improvement rate of the 60 patients was 71.7% (43/60). After treatment, the visual acuity improvement rate of the study group was 83.3% (25/30), which was significantly higher than that of the control group (60.0%, 18/30), and the difference was statistically significant (*χ*^2^ = 4.022, *P*=0.045, Table 3).

### 3.4. Treatment Effect of Patients

After neuroendoscopic endonasal transsphenoidal surgeries, the significant effective rate, effective rate, and ineffective rate were 66.7% (20/30), 30.0% (9/30), and 3.3% (1/80), respectively. In the control group, the significant effective rate, effective rate, and ineffective rate were 36.7% (11/30), 46.7% (14/30), and 16.7% (5/30), respectively. The total effective rate of the study group was 96.7% (29/30), which was significantly higher than that of the control group (83.3%, 25/30), and the difference was statistically significant (*χ*^2^ = 6.367, *P*=0.041), as shown in Table 4.

### 3.5. Postoperative Adverse Reactions

Anosmia, headache, intracranial infection, and cerebrospinal fluid leakage occurred in 2, 3, 1, and 4 patients, respectively, in the study group. In the control group, olfactory dysfunction, headache, intracranial infection, and cerebrospinal fluid leakage occurred in 3, 3, 1, and 2 patients, respectively. The total incidence of adverse events in the study group was 33.3% (10/30), which was like that in the control group (30.0%, 9/30) without significant difference (*χ*^2^ = 0.077, *P*=0.781), as shown in Table 5.

## 4. Discussion

In this study, compared with the control group, neuroendoscopic endonasal transsphenoidal surgeries for tuberculum sellae meningioma can increase the total resection rate of tumor and improve visual impairment and treatment effect. Notably, neuroendoscopic endonasal transsphenoidal surgeries did not increase the incidence of adverse events.

Epidemiological studies suggest that tuberculum sellae meningioma (TSM) accounts for 3% to 10% of intracranial meningiomas, with some age and gender differences [9]. Compared with meningiomas in other parts, tuberculum sellae meningiomas have their own characteristics. The main manifestations of tuberculum sellae meningiomas are visual impairment and visual field impairment, which may be accompanied by headache and endocrine abnormalities [10]. At present, surgical resection is the main method for the treatment of tuberculum sellae meningioma, but due to the deep tumor site, delicate and complex surrounding anatomical structure, and other reasons, the surgical risk is high, and the postoperative effect is not good [11]. Improving postoperative visual acuity is a major difficulty in surgical treatment, and the reasons affecting postoperative visual acuity recovery include patient age, concomitant diseases, tumor size, tumor blood supply, and degree of resection [11].

Intracranial endoscopic pterional approach is a relatively mature operation in clinical practice and is the standard surgical treatment for tuberculum sellae meningioma. The study suggested that the intracranial endoscopic pterional approach for tuberculum sellae meningioma resection had the following problems. For example, the total tumor resection rate and visual acuity improvement rate are not satisfactory, the brain tissue is pulled more during the operation, the wound surface is larger, the operation time is longer, other problems make the postoperative recovery of patients slow, and various postoperative complications may occur [6]. Neuroendoscopic endonasal transsphenoidal surgeries are a newly developed surgical method in recent years, which has been gradually applied in clinical practice and can effectively solve the above problems. In this study, neuroendoscopic endonasal transsphenoidal surgeries for tuberculum sellae meningioma were found to have a higher tumor resection rate (93.3% vs 70%) and visual acuity improvement rate (83.3% vs 60.0%) than intracranial endoscopic pterional approach. Similar to our study, previous studies also found that the total resection rate and visual recovery rate of neuroendoscopic endonasal transsphenoidal surgeries were higher than that of the intracranial endoscopic pterional approach [12]. Neuroendoscopic endonasal transsphenoidal surgeries for the treatment of tuberculum sellae tumors are a hotspot in the field of neurosurgery. The key technique is to remove the sphenoid plateau and tuberculum sellae and expose the suprasellar region and optic chiasma [13].

Previous studies have suggested that neuroendoscopic endonasal transsphenoidal surgeries may increase the risk of postoperative cerebrospinal fluid leakage and other adverse reactions [14]. However, in this study, neuroendoscopic endonasal transsphenoidal surgeries did not increase the risk of adverse reactions compared to the intracranial endoscopic transpteral approach (33.3% vs 30%, *P* > 0.05). This may be mainly explained as follows: The neuroendoscopic endonasal transsphenoidal surgeries can provide a good visual angle and clear surgical field, especially with obvious advantages in protecting optic chiasma and nourishing blood vessels [15]. In addition, studies have suggested that the incidence of cerebrospinal fluid leakage can be significantly reduced with adequate sellar floor repair techniques [16].

In addition to age and gender, duration of visual impairment and the relationship between tumor and optic chiasma and optic nerve were also important factors affecting postoperative visual recovery. In this study, there was no significant difference in the above factors between the two groups. Therefore, for patients with tuberculum sellae meningioma, the neuroendoscopic endonasal transsphenoidal surgeries may have a protective effect independent of the above factors. Determining the optimal approach is a nuanced process that must account for patient and tumor characteristics as well as surgeon preference and skill in order to achieve the best outcome for each individual patient [17]. The most important outcomes, and goals of surgery, are improving/preserving visual function, maximizing the extent of resection and minimizing infection and cerebrospinal fluid leak [17].

It should be reminded that this study has limitations such as small sample size, short study time and few collection factors. Future long-term follow-up studies with a large sample size are needed to further validate the advantages of neuroendoscopic endonasal transsphenoidal surgeries in patients with tuberculum sellae meningioma.

In conclusion, neuroendoscopic endonasal transsphenoidal surgeries have significant efficacy and significantly improve the visual acuity of patients without increasing adverse reactions, which is worthy of clinical promotion.

## Figures and Tables

**Table 1:** Comparison of general data and clinical features of tuberculum sellae meningioma patients in two groups.

	Study group	Control group	*t*/*χ*^2^	*P* value
Case	30	30	—	—
Age, years	54.8 ± 9.8	56.8 ± 8.2	−0.859	0.394
Sex, *n* (%)			2.500	0.114
Male	15 (50.0)	9 (30.0)		
Female	15 (50.0)	21 (70.0)		
Duration of visual impairment, months	15.7 ± 4.3	15.1 ± 4.0	0.559	0.579
Duration of headache, months	5.5 ± 3.7	5.7 ± 3.5	−0.180	0.858
Hypertension, *n* (%)	18 (60.0)	16 (53.3)	0.271	0.602
Diabetes mellitus, *n* (%)	6 (20.0)	10 (33.3)	1.364	0.243
Coronary heart disease, *n* (%)	5 (16.7)	4 (13.3)	0.131	0.718
Systolic blood pressure, mmHg	133.8 ± 13.9	135.8 ± 12.6	−0.604	0.548
Diastolic blood pressure, mmHg	87.7 ± 12.6	85.2 ± 15.9	0.666	0.508
Tumor diameter, (cm)	2.6 ± 0.5	2.7 ± 0.3	−1.643	0.106
Squeezing optic chiasm, *n* (%)	6 (20.0)	9 (30.0)	0.800	0.371
Relation with optic nerve, *N* (%)			0.375	0.829
Elation	14 (46.7)	13 (43.3)		
Adhesion	6 (20.0)	8 (26.7)		
Circumference	10 (33.3)	9 (30.0)		

**Table 2:** Comparison of tumor resection between the two groups^*∗*^.

Groups	Degree of tumor resection		Total
	Total ectomy	Subtotal ectomy	
Study group	28	2	30
Control group	21	9	30
Total	49	11	60

^*∗*^ *χ* ^2^ = 5.455, *P*=0.020.

**Table 3:** Comparison of visual improvement between the two groups^*∗*^.

Groups	Vision improvement		Total
	Improvement	Nonimprovement	
Study group	25	5	30
Control group	18	12	30
Total	43	17	60

^*∗*^ *χ* ^2^ = 4.022, *P*=0.045.

**Table 4:** Comparison of therapeutic effects between the two groups during three months after surgery.

	Case	Significantly effective, *n* (%)	Effective, *n* (%)	Ineffective, *n* (%)	Total effective rate, (%)
Study group	30	20 (66.7)	9 (30.0)	1 (3.3)	96.7
Control group	30	11 (36.7)	14 (46.7)	5 (16.7)	83.3

*χ* ^2^	6.367				
*P* value	0.041				

**Table 5:** Comparison of postoperative adverse reactions between the two groups.

	Anosmia, *n* (%)	Headache, *n* (%)	Intracranial infection, *n* (%)	Cerebrospinal fluid leakage, *n* (%)	Total adverse reactions, *n* (%)
Study group	2 (6.7)	3 (10.0)	1 (3.3)	4 (13.3)	10 (33.3)
Control group	3 (10.0)	3 (10.0)	1 (3.3)	2 (6.7)	9 (30.0)

*χ* ^2^	0.077				
*P* value	0.781				

## Data Availability

The data used to support the findings of this study are available from the corresponding author upon request.
